# Maternal diabetes up‐regulates NOX2 and enhances myocardial ischaemia/reperfusion injury in adult offspring

**DOI:** 10.1111/jcmm.13500

**Published:** 2018-01-29

**Authors:** Lili Zhang, Xiaoyan Wang, Yan Wu, Xiangru Lu, Peter Chidiac, Guoping Wang, Qingping Feng

**Affiliations:** ^1^ Institute of Pathology Tongji Hospital Tongji Medical College Huazhong University of Science and Technology Wuhan China; ^2^ Department of Physiology and Pharmacology Schulich School of Medicine and Dentistry University of Western Ontario London Ontario Canada; ^3^ Department of Metabolism and Endocrinology The Second Xiangya Hospital Central South University Changsha China

**Keywords:** maternal diabetes, NOX2, reactive oxygen species, myocardial ischaemia and reperfusion injury, mTOR, developmental origins of health and disease

## Abstract

Offspring of diabetic mothers are at risk of cardiovascular diseases in adulthood. However, the underlying molecular mechanisms are not clear. We hypothesize that prenatal exposure to maternal diabetes up‐regulates myocardial NOX2 expression and enhances ischaemia/reperfusion (I/R) injury in the adult offspring. Maternal diabetes was induced in C57BL/6 mice by streptozotocin. Glucose‐tolerant adult offspring of diabetic mothers and normal controls were subjected to myocardial I/R injury. Vascular endothelial growth factor (VEGF) expression, ROS generation, myocardial apoptosis and infarct size were assessed. The VEGF‐Akt (protein kinase B)‐mammalian target of rapamycin (mTOR)‐NOX2 signalling pathway was also studied in cultured cardiomyocytes in response to high glucose level. In the hearts of adult offspring from diabetic mothers, increases were observed in VEGF expression, NOX2 protein levels and both Akt and mTOR phosphorylation levels as compared to the offspring of control mothers. After I/R, ROS generation, myocardial apoptosis and infarct size were all significantly higher in the offspring of diabetic mothers relative to offspring of control mothers, and these differences were diminished by *in vivo* treatment with the NADPH oxidase inhibitor apocynin. In cultured cardiomyocytes, high glucose increased mTOR phosphorylation, which was inhibited by the PI3 kinase inhibitor LY294002. Notably, high glucose‐induced NOX2 protein expression and ROS production were inhibited by rapamycin. In conclusion, maternal diabetes promotes VEGF‐Akt‐mTOR‐NOX2 signalling and enhances myocardial I/R injury in the adult offspring. Increased ROS production from NOX2 is a possible molecular mechanism responsible for developmental origins of cardiovascular disease in offspring of diabetic mothers.

## Background

The developmental origins of health and disease theory are based on evidence that nutritional, hormonal and metabolic factors during early life from preconception to childhood have a lifelong impact on adult health and disease 1, 2. For example, intrauterine exposure to hyperglycaemia has been shown to cause permanent foetal changes and increase susceptibility to a number of chronic problems including cardiovascular and metabolic diseases in adult life 3, 4, 5, 6, 7. Additionally, patients with diabetes have an increased risk of cardiovascular morbidity and mortality, and the diabetic heart is prone to ischaemic injury 8, 9. However, the underlying molecular mechanisms are not well understood.

Reactive oxygen species (ROS) are a hallmark of cardiovascular disease 10 and have been shown to play a key role in myocardial ischaemia and reperfusion (I/R) injury 11, 12. In cardiac tissues, NADPH oxidases (NOX) are the major source of ROS under both physiological and pathological conditions 12, 13, 14. The NOX family has seven members, NOX1‐5, Duox1 and Duox2 with NOX2 being the predominant isoform in the heart. Activation of cardiomyocyte NOX2 contributes to cardiac injury after myocardial infarction 14, 15, 16, 17. Notably, high glucose levels induce NOX2 activation in cultured cardiomyocytes 18, 19. However, whether maternal diabetes up‐regulates myocardial NOX2 expression in the adult offspring and what signalling pathway may lead to its up‐regulation are not known. Furthermore, the role of NADPH oxidase in I/R injury in the diabetic offspring remains to be elucidated.

The mammalian target of rapamycin (mTOR) is a serine/threonine protein kinase and functions through two multiprotein complexes, mTOR complex 1 (mTORC1) and mTORC2 20. Serving as an nutrient/energy/redox sensor, activated mTORC1 promotes protein synthesis while mTORC2 regulates metabolism, cell proliferation and cytoskeleton organization. Notably, growth factors activate mTOR *via* phosphatidylinositide 3‐kinase (PI3K)/Akt signalling to increase protein synthesis 20. Importantly, vascular endothelial growth factor (VEGF) is a major growth factor, which is up‐regulated in the foetal heart during maternal diabetes 21, 22. However, changes in Akt/mTOR signalling in the glucose‐tolerant adult offspring of maternal diabetes are not well understood. This study was aimed to test the hypothesis that prenatal exposure to maternal diabetes up‐regulates myocardial NOX2 expression *via* Akt/mTOR signalling and enhances I/R injury in the glucose‐tolerant adult offspring in mice.

## Materials and methods

### Animals

C57BL/6 wild‐type mice were purchased from Jackson Laboratory (Bar Harbor, Maine). Animals in this study were handled in accordance with the *Guide for the Care and Use of Laboratory Animals*, published by the U.S. National Institutes of Health (8th edition, 2011). Use of animals was approved by the Animal Care Committee at the University of Western Ontario, Canada.

### Induction of maternal diabetes

Adult female mice were treated with streptozotocin (STZ, 50 mg/kg per day, IP, for 4 consecutive days) as in our recent studies 21, 23. Non‐fasting blood glucose levels were measured 1 week after the final STZ injection with a glucose meter (OneTouch Ultra2, LifeScan, Burnaby, BC, Canada). Female mice with blood glucose levels higher than 11 mmol/l were bred to normal males to generate offspring for *in vivo* studies. Controls were produced by breeding normal males to females that had not received STZ treatment. Non‐fasting blood glucose levels were also measured between embryonic day 15.5 and 18.5. The number of neonates per mother was not fixed.

### Intraperitoneal glucose tolerance test (IPGTT)

Adult male offspring (3–6 months old) from control and diabetic mothers were fasted for 16 hrs and treated with D‐glucose at 2 g/kg, IP. Blood glucose was measured at 0, 30, 60, 90 and 120 min. after glucose administration.

### Induction of myocardial I/R

The adult male offspring (3–6 months old) from control and diabetic mothers were subjected to sham surgery, myocardial I/R or I/R + apocynin (NADPH oxidase inhibitor) for a total of six groups (*n *=* *6 per group). Briefly, the adult male offspring were anaesthetized with ketamine (50 mg/kg, i.p.) and xylazine (12.5 mg/kg, i.p.). The adequacy of anaesthesia was confirmed by the absence of withdrawal reflex to tail pinch. Subsequently, mice were intubated and artificially ventilated with a respirator (SAK‐830, CWE, Ardmore, PA). The left descending coronary artery was occluded by an 8‐0 suture around it with a PE‐50 tube. After 45 min., the tube was removed to allow reperfusion for either 1 or 3 hrs for measurements of ROS generation and infarct size, respectively 24, 25. To study the effect of NADPH oxidase inhibition, some mice were treated with saline (vehicle) or apocynin (10 mg/kg, IP) for 30 min. before induction of myocardial ischaemia.

### Infarct size measurement

Infarct size was determined as described previously 25, 26. In brief, after 45 min. of ischaemia and 3 hrs of reperfusion (I/R), the left coronary artery was re‐occluded using the same suture. Mice were killed by ketamine overdose. The heart was isolated and perfused through the ascending aorta with Evans blue dye (1%, 0.7 ml) to determine the non‐ischaemic (perfused, blue) and ischaemic (not perfused, not blue) areas of the heart. Then, the heart was sectioned into four pieces and stained with 1% triphenyltetrazolium chloride (TTC) for 10 min. at room temperature. The viable, ischaemic tissue was stained into a red colour, while infarct area was unstained (white colour). Each heart section was photographed and weighed. The weight of non‐risk (blue), infarcted (white) and at‐risk areas (not blue) was calculated. Infarct size was measured as percentage of the weight of infarct area relative to the area at risk 25, 26.

### Analysis of superoxide generation

Superoxide generation in the myocardium and cultured cardiomyocytes was determined using dihydroethidium (DHE, Invitrogen, Carlsbad, CA, USA) staining 27. Briefly, frozen sections (10 μm) of the LV myocardium were treated with DHE (2 μM) with and without diphenyleneiodonium (DPI, 30 μM) at 37°C for 30 min. in a dark, humidified chamber. DHE red fluorescence was imaged at ×400 magnification using a fluorescence microscope (Observer D1, Zeiss, Germany) connected to a digital camera. The fluorescent signal intensities were analysed and quantified using AxioVision software (Zeiss).

### Neonatal mouse cardiomyocyte culture

Neonatal cardiomyocytes were cultured as previously described 28. Briefly, neonatal mouse hearts were isolated and minced in bicarbonate, Ca^2+^‐ and Mg^2+^‐free Hanks balanced salt solution. Cardiomyocytes were dispersed by incubation with 22.5 μg/ml liberase 4 (Roche, Laval, Quebec) in D‐Hanks at 37°C with gentle agitation for 10 min. After centrifugation at 200 *g* for 5 min., cells were collected and resuspended in FCS‐containing M199 medium. After 1 hr of pre‐plating, non‐cardiomyocytes were removed. Cardiomyocytes were plated in M199 medium containing 10% foetal bovine serum on culture plates pre‐coated with 1% gelatin. Neonatal cardiomyocytes were treated with high glucose (25 mM D‐glucose) or normal glucose (5 mM D‐glucose + 20 mM L‐glucose) in the presence or absence of rapamycin (5 nM, Cell Signaling Technology) and LY294002 (10 μM).

### Western Blot analysis

Protein samples from tissue homogenates or cell lysates were subjected to separation on a 10% SDS‐PAGE gel, followed by electrotransfer to nitrocellulose membranes. Blots were probed with specific antibodies against NOX2, cytochrome c (BD Bioscience, San Jose, CA, USA), VEGF‐A (Chemicon International, Temecula, CA, USA), GAPDH (Dallas, TX, USA), α‐actinin (Sigma‐Aldrich, St. Louis, MO, USA), phospho‐Akt (Ser473), total Akt, phospho‐mTOR (Ser2448) and total mTOR (Cell Signaling, Danvers, MA, USA), respectively. Signals were detected by the enhanced chemiluminescence detection method and quantified by densitometry using FluorChem 8000 software (Alpha Innotec, San Leandro, CA, USA).

### Real‐time RT‐PCR

Total RNA was extracted from mouse hearts and cultured neonatal cardiomyocytes using TRIzol (Invitrogen) as per manufacturer's instructions. Total RNA (1 μg) was used to synthesize cDNA using Moloney murine leukaemia virus reverse transcriptase. The oligonucleotide primer sequences for NOX2 were 5′ TGT ACT GTC CCA CCT CCA TCT 3′ (forward) and 5′ GCT GGA AAC CCT CCT ATG ACT 3′ (reverse). Primers for VEGF‐A, bFGF, IGF‐1 and 28S were the same as our previous articles 26, 29. Quantitative real‐time PCR was conducted using EvaGreen qPCR MasterMix (Applied Biological Materials, Vancouver, BC, Canada). Values were compared to that of 28S rRNA, and the relative expression of these genes was obtained.

### Assessment of myocardial apoptosis

Myocardial apoptosis was assessed using caspase‐3 activity and cytosolic DNA fragments assays 29, 30. Caspase‐3 activity was determined using a QuantiZyme Assay System (Biomol, Plymouth Meeting, PA, USA). Briefly, heart tissues were homogenized and protein concentrations were determined. Samples (50 μg protein) were incubated at 37°C for 16 hrs in the presence of caspase‐3 substrate acetyl Asp‐Glu‐Val‐Asp 7‐amido‐4‐methylcoumarin (Ac‐DEVD‐AMC) with and without the inhibitor *N*‐acetyl‐Asp‐Glu‐Val‐Asp‐al (Ac‐DEVD‐CHO). Fluorescence intensity (excitation at 355, emission at 405) was measured using a multilabel plate reader (SpectraMax M5, Molecular Devices, Sunnyvale, CA, USA). Data are expressed as the amount of AMC substrate cleaved/μg protein. Cytosolic DNA fragments were determined using a Cell Death Detection ELISA kit (Roche, Mississauga, ON, USA) as we previously described 29, 30.

### Reagents

Ketamine and xylazine were purchased from Bioniche Animal Health Canada Inc. (Belleville, ON, USA) and Bachem AG, Switzerland, respectively. All other reagents if unspecified were obtained from Sigma‐Aldrich, St. Louis, MO, USA.

### Statistical analysis

Data are presented as mean ± S.E.M. Results were analysed using one‐ or two‐way ANOVA followed by Newman–Keuls or Bonferroni *post hoc* test for multigroup comparisons. Unpaired Student's Test was used for comparisons between two groups. Neonatal mortality was analysed by chi‐square test. *P *<* *0.05 was considered statistically significant.

## Results

### Myocardial NOX2 protein is up‐regulated in offspring of diabetic mothers

Maternal diabetes increases the risk of developing congenital heart defects (CHDs) in the foetus by five‐ to 10‐fold 31. Our recent studies have shown that high blood glucose levels (>25 mmol/l) during pregnancy induced by STZ (80 mg/kg, i.p. for 3 days) result in CHDs in the offspring 21, 23. In this study, a milder STZ dosing protocol (50 mg/kg i.p. for 4 days) was used to induce maternal diabetes, with significantly higher non‐fasting blood glucose levels than non‐diabetic controls at embryonic day 15.5–18.5 (Fig. 1A, *P* < 0.01). However, most pregnant mice (11 of 14) had blood glucose levels lower than 25 mmol/l and no apparent CHDs were observed in any of the offspring of diabetic mothers.

**Figure 1:** Myocardial NOX2 protein levels are up‐regulated in adult offspring of diabetic mothers (ODM). **A**, Non‐fasting blood glucose levels in control (*n *=* *9) and diabetic mothers (*n *=* *14) during pregnancy at embryonic day 15.5–18.5. **B**, Intraperitoneal glucose tolerance test (IPGTT) results were not significantly different between adult offspring of control mothers (OCM) and ODM. **C**, Myocardial NOX2 protein expression was analysed by Western blotting in the adult OCM and ODM. Real‐time PCR analysis for myocardial RNA levels of NOX2 (**D**) and NOX4 (**E**) in the adult OCM and ODM. Data are mean ± S.E.M., *N *=* *4–8 mice per group, *P <* *0.05 *versus* OCM, **P <* *0.01 *versus* control mothers.

Litter size at birth was significantly smaller in the diabetic group compared with normal controls (*P *<* *0.05; Table 1). However, neonatal mortality and the body weights of pups were similar between the two groups. After weaning, the pups of the two groups were fed with the same diet. Body weight at 3–4 months of age was not significantly different between the two groups. The offspring of diabetic mothers were hyperphagic compared control counterparts (*P *<* *0.05). However, water consumption was not significantly different between the two groups (Table 1).

**Table 1:** General characteristics of offspring of control mice and diabetic mothers

Parameters	Offspring of control mothers	Offspring of diabetic mothers
Litter size	9.6 ± 0.8 (12)	7.0 ± 0.7 (12)^a^
Neonatal mortality (dead/total)	1.72% (2/116)	3.57% (3/84)
Neonatal body weight (g)	1.27 ± 0.03 (24)	1.20 ± 0.03 (30)
Body weight at 3–4 months (g)	27.16 ± 0.73 (12)	28.86 ± 0.88 (12)
Food intake at 2 months (g/g body weight/24 hrs)	0.16 ± 0.01 (10)	0.20 ± 0.01 (6)^a^
Water intake at 2 months (ml/g body weight/24 hrs)	0.30 ± 0.02 (10)	0.29 ± 0.02 (6)

Data are mean ± S.E.M. except for neonatal mortality. Unpaired Students test was used for comparisons between two groups. Neonatal mortality was analysed by chi‐square test.

a *P *<* *0.05 *versus* control. Mouse numbers are in brackets.

To assess if the adult male offspring (3–6 months old) of diabetic mothers have glucose intolerance, IPGTT was performed. Our results show that there was no significant difference in glucose tolerance between the offspring of control and diabetic mothers (Fig. 1B). NOX2 is the predominant isoform of NADPH oxidase in the heart and a main source of ROS generation 12. We thus examined NOX2 expression in the heart under basal physiological conditions. Western blot analysis shows that myocardial NOX2 protein levels were significantly up‐regulated in adult offspring of diabetic mothers compared to those of control mothers (Fig. 1C). However, qPCR results showed no significant difference in NOX2 mRNA expression between the two groups (Fig. 1D), suggesting that up‐regulation of NOX2 protein in diabetic offspring may involve mechanisms independent of gene transcription. Additionally, the mRNA levels of NOX1 and NOX4 were examined. Our data show that myocardial NOX4 mRNA expression was not significantly altered between the two groups (Fig. 1E), while NOX1 mRNA was not detectable up to 32 cycles of qPCR amplification in the adult heart.

### Offspring of diabetic mothers are susceptible to I/R injury *via* ROS generation

To study susceptibility to I/R injury, the adult offspring of diabetic mothers and normal control mothers were subjected to 45 min. of ischaemia followed by 1 or 3 hrs of reperfusion. Results show that myocardial ROS generation assessed using DHE staining was significantly higher in the offspring of diabetic mothers compared to those of control mothers (Fig. 2A and B). Infarct size was assessed using Evans blue and TTC staining. Our data show a larger infarct size in the diabetic offspring, while area at risk was not significantly changed (Fig. 2C and D). Notably, *in vivo* treatment with the NADPH oxidase inhibitor apocynin significantly decreased ROS generation and infarct size in the offspring of diabetic mothers (Fig. 2B and D). To assess myocardial apoptosis, cytosolic cytochrome c levels, caspase‐3 activity and cytosolic DNA fragments were determined. Our results show that I/R increased caspase‐3 activity and cytosolic levels of cytochrome c and DNA fragments in the myocardium and that these were all significantly higher in the offspring of diabetic mothers (Fig. 3A–C). Furthermore, treatment with apocynin *in vivo* significantly reduced all three apoptotic parameters in the offspring of diabetic mothers (Fig. 3A–C). These data suggest that the offspring of diabetic mothers are more susceptible to myocardial I/R injury *via* ROS generation from NADPH oxidase.

**Figure 2:** The adult offspring of diabetic mothers (ODM) are more susceptible to myocardial I/R injury. Adult male mice were subjected to sham or I/R (45 min. of ischaemia followed by 1 hr (**A** and **B**) or 3 hrs (**C** and **D**) of reperfusion). Some mice were treated with apocynin (10 mg/kg, IP) before ischaemia (I/R + apocynin). **A** and **B**, Myocardial superoxide generation after I/R with and without apocynin treatment was assessed in the adult offspring of control mothers (OCM) and ODM by DHE staining. **C** and **D**, Infarct size after I/R with and without apocynin treatment. Data are mean ± S.E.M. *N *=* *6 mice per group. *P <* *0.05 *versus* respective sham in B or I/R OCM in D; ^†^ *P *<* *0.05 *versus* respective OCM in B or I/R ODM in D; ^#^ *P *<* *0.05 *versus* I/R ODM in B.

**Figure 3:** Myocardial apoptosis after I/R in offspring of control (OCM) and diabetic mothers (ODM). Adult male mice were subjected to 45 min. of ischaemia followed by 3 hrs of reperfusion (I/R). Some mice were treated with apocynin (10 mg/kg, IP) before ischaemia. **A**, Western blot analysis of cytosolic cytochrome c levels in the myocardium. **B** and **C**, Myocardial apoptosis measured by cytosolic DNA fragments and caspase‐3 activity. Data are mean ± S.E.M. *N *=* *4–5 mice per group. *P <* *0.05 *versus* respective sham; ^†^ *P *<* *0.05 *versus* I/R OCM; ^#^ *P *<* *0.05 *versus* I/R ODM.

### VEGF/Akt/mTOR signalling is increased in offspring of maternal diabetes

mTOR is a central regulator of protein synthesis 32. To address the mechanism by which NOX2 protein expression was up‐regulated, we examined growth factor/Akt/mTOR signalling pathway in the hearts of the offspring of diabetic mothers. Real‐time RT‐PCR analysis showed that myocardial VEGF‐A mRNA levels were significantly higher in the offspring of diabetic compared to those of control mothers (Fig. 4A, *P* < 0.05) while bFGF and IGF‐1 mRNA levels were not significantly different between the two groups (Fig. 4B and C, P = n.s.). Western blot analysis showed that VEGF‐A protein levels were also significantly higher in the offspring of diabetic compared to those of control mothers (Fig. 4D, *P* < 0.05). Furthermore, phosphorylation of Akt and mTOR was significantly increased in the hearts of offspring of diabetic mothers compared to control counterparts (Fig. 4E and F, *P* < 0.05). These results suggest that activity of the Akt/mTOR signalling pathway is increased in the hearts of offspring of diabetic mothers, causing higher NOX2 protein expression.

**Figure 4:** Increased VEGF/Akt/mTOR signalling in adult offspring of diabetic mothers (ODM). **A–C**, Myocardial mRNA levels of VEGF‐A, bFGF and IGF‐1 in the adult offspring of control mothers (OCM) and ODM. **D–F**, Western blot analysis of myocardial VEGF‐A, phosphorylation of Akt and mTOR protein levels in the adult OCM and ODM. Data are mean ± S.E.M., *N *=* *4–5 mice per group, *P <* *0.05 compared to OCM.

### High glucose induces NOX2 expression *via* Akt/mTOR signalling in cardiomyocytes

To further examine changes in Akt/mTOR signalling in NOX2 protein expression, primary cultures of neonatal mouse cardiomyocytes were employed to mimic cardiomyocyte exposure to hyperglycaemia *in utero*. After cellular exposure to high glucose (25 mM) for 4 days, VEGF‐A mRNA and protein levels were significantly up‐regulated (Fig. 5A and B, *P* < 0.05). Consistent with mTOR activation in the myocardium of adult diabetic offspring, high glucose treatment significantly increased mTOR phosphorylation, which was blocked by rapamycin (5 nM) (Fig. 5C, *P* < 0.05) and by the PI3 kinase inhibitor LY294002 (10 μM) (Fig. 5D, *P* < 0.05). Notably, high glucose also resulted in significantly higher NOX2 protein levels in cardiomyocytes compared with normal glucose (5 mM) controls, and this effect was completely blocked by an mTOR inhibitor rapamycin (5 nM) (Fig. 6A and B, *P* < 0.05). To assess NADPH oxidase activity in cultured cardiomyocytes, ROS generation was determined by dihydroethidine (DHE) staining. Our data show that high glucose significantly increases ROS generation and that this is completely blocked by rapamycin (Fig. 6C and D, *P* < 0.05). Taken together, these results demonstrate that high glucose induces NOX2 protein expression in cardiomyocytes through activation of the Akt/mTOR signalling pathway.

**Figure 5:** High glucose (HG) induces VEGF/Akt/mTOR signalling in cultured neonatal mouse cardiomyocytes. **A** and **B**, VEGF‐A mRNA and protein levels in cultured cardiomyocytes analysed by real‐time PCR and ELISA, respectively. **C** and **D**, Western blot analysis of mTOR phosphorylation in cultured cardiomyocytes. **C**, HG‐induced mTOR phosphorylation was blocked by PI3 kinase inhibitor LY294002. **D**, HG‐induced mTOR phosphorylation was inhibited by rapamycin. Data represent mean ± S.E.M., *N *=* *3 per group, *P <* *0.05 compared to normal glucose (NG) group, † < 0.05 compared to HG vehicle group.

**Figure 6:** High glucose (HG) induces NOX2 expression and superoxide generation in cultured cardiomyocytes *via* mTOR. **A** and **B**, Western blot analysis of NOX2 protein levels in cultured neonatal mouse cardiomyocytes with GAPDH as a loading control. **C** and **D**, Analysis of superoxide generation in cultured cardiomyocytes using dihydroethidine (DHE) staining. Data are mean ± S.E.M., *N *=* *3 per group, *P <* *0.05 compared to normal glucose (NG) group, † < 0.05 compared to HG vehicle group.

## Discussion

The major findings of the present study are that myocardial NOX2 protein levels and ROS production were higher and that the VEGF/Akt/mTOR signalling pathway was activated in the normal glycemic and glucose‐tolerant offspring of diabetic mothers compared to normal controls. Following myocardial I/R, myocardial apoptosis and infarct size were significantly increased in the offspring of diabetic mothers, changes which were diminished by treatment with the NADPH oxidase inhibitor apocynin. In cultured neonatal cardiomyocytes, high glucose activated mTOR, which was blocked by the PI3‐kinase inhibitor LY294002. Furthermore, increases in NOX2 protein levels and ROS generation in cardiomyocytes induced by high glucose were inhibited by rapamycin, the prototype mTOR inhibitor. Our results suggest NOX2 protein expression is up‐regulated in the offspring of diabetic mothers through the VEGF/Akt/mTOR pathway, and the normal glycemic offspring of diabetic mothers are susceptible to myocardial I/R injury, which is mediated by ROS generation from NADPH oxidase (Fig. 7).

**Figure 7:** Proposed signalling pathway of maternal diabetes leading to NOX2 expression and cardiac I/R injury in the adult offspring.

Diabetes is one of the major health concerns worldwide. Increasing evidence shows that children born from diabetic pregnancy are at a higher risk of cardiovascular and metabolic morbidity in their adulthood 4, 33, 34, 35. However, the underlying mechanisms are not fully understood. As maternal glucose freely crosses the placenta, offspring of diabetic mothers are exposed to high blood glucose levels during gestation 3. Studies in cultured adult cardiomyocytes have shown that high glucose increases the expression of NOX2 36, the predominant isoform of NADPH oxidase in heart. However, it is not known if maternal diabetes up‐regulates myocardial NOX2 expression in normal glycemic and glucose‐tolerant offspring. In the present study, we tested the hypothesis that maternal diabetes up‐regulates NOX2 expression and enhances cardiac I/R injury in the adult offspring. The offspring of diabetic mothers were generated from female mice treated with low dose STZ before they were mated with normal males. Notably, the offspring of diabetic mothers at 3–6 months of age had normal blood glucose levels and did not exhibit any glucose intolerance. However, these mice exhibited significantly higher NOX2 protein expression without any changes in its mRNA levels in the heart. Of note, high glucose has been shown to promote protein synthesis 37, 38. As mTOR is a central regulator of protein synthesis in response to stress and growth factor stimulations and regulated by PI3K/Akt 20, we investigated the role of PI3K/Akt/mTOR signalling pathway in the present study. Our data showed that mTOR phosphorylation was increased in cardiomyocytes in response to high glucose treatment and blocked by the PI3K inhibitor LY294002. Furthermore, increased NOX2 expression induced by high glucose was inhibited by rapamycin, suggesting that up‐regulation of NOX2 protein levels is mediated *via* the PI3K/Akt/mTOR signalling pathway. Hyperglycaemia promotes expression and release of VEGF 39, 40, which activates the PI3K/Akt/mTOR signalling pathway 20. We recently showed that VEGF mRNA levels are increased in the foetal hearts in the presence of maternal diabetes 21. In agreement with this notion, we now show that VEGF expression is increased in the hearts of offspring of diabetic mothers and in high glucose‐treated cardiomyocytes and that this is associated with activation of the PI3K/Akt/mTOR signalling pathway.

ROS have been shown to play a pivotal role in myocardial I/R injury 11, 12. Excessive production of ROS leads to oxidation and damage of membranes and macromolecules, which accelerates cell death through apoptosis and necrosis. On the other hand, maternal treatment with melatonin, which has antioxidant properties, has been shown to decrease cardiac I/R injury in adult mouse offspring that are glucose intolerant 41. Additionally, both ROS and apoptosis are increased in T cells of hyperglycaemic offspring of diabetic mothers 42. However, NOX2 expression and its role in the offspring of diabetic mothers are not clear. In the present study, we show that myocardial NOX2 protein levels were up‐regulated in normoglycemic and glucose‐tolerant adult offspring of diabetic mothers. In response to myocardial I/R, the offspring of diabetic mothers exhibited higher infarct size compared to controls, indicating enhanced I/R injury. Furthermore, ROS generation and apoptosis were also increased in the hearts of offspring of diabetic mothers. These changes were all inhibited by *in vivo* treatment of apocynin, an NADPH oxidase inhibitor, suggesting a critical role of NOX2 in enhanced cardiac injury in the offspring of diabetic mothers.

## Conclusion

Maternal diabetes up‐regulates myocardial NOX2 protein expression in normoglycemic and glucose‐tolerant adult offspring. Up‐regulation of NOX2 is associated with activation of the VEGF/Akt/mTOR signalling pathway. Increased NOX2 protein expression results in ROS production and myocardial apoptosis, leading to enhanced I/R injury in the offspring of diabetic mothers (Fig. 7). Recent studies have shown that increased NOX2 activity is associated with cardiac injury, endothelial dysfunction, atherosclerosis and islet β‐cell injury 17, 43, 44. The findings of the present study suggest that up‐regulation of NOX2 expression and activity is likely a molecular mechanism responsible for the developmental origins of cardiovascular disease in the offspring of diabetic mothers, providing a new hypothesis that could be tested in future clinical studies.

## Conflict of interest

The authors declare no conflict of interest.
